RETRACTED

# Study on the Evaluation of Lung Cancer Patients from the Three Aspects of Emotion

**DOI:** 10.1155/2022/8139680

**Published:** 2022-09-15

**Authors:** Panpan Li, Jiangli Yu, Xiaohui Wang, Xiaonan Pang, Chengjing Yu, Yingqiong Xu

**Affiliations:** ^1^Department of Pulmonary and Critical Care Medicine, The Sixth Medical Center of PLA General Hospital, Beijing 100048, China; ^2^Department of Neurology, The Second Medical Center & National Clinical Research Center for Geriatric Diseases, Chinese PLA General Hospital, Beijing 100048, China; ^3^Department of Oncology, The Second Affiliated Hospital of Anhui Medical University, Hefei 230088, China

## Abstract

In recent years, epidemiological survey data have shown that lung cancer is the tumor with the fastest increase in cancer incidence and mortality in China. The incidence and mortality of lung cancer in China rank first among tumors, and 80% of patients die within one year of diagnosis. This paper aims to study the evaluation of lung cancer patients from three aspects of emotion, coping style, and Quality of Life (QoL), expounding on the changes in emotion, coping style, and QoL in lung cancer patients after chemotherapy. We assess the negative emotions and survival of lung cancer patients after chemotherapy quality satisfaction survey research. We investigate the general data, QoL, and coping styles of 219 lung cancer patients undergoing chemotherapy before, during, and after chemotherapy based on the artificial intelligence processor. All survey data are input into SPSS 19 for descriptive and relevant statistical analysis. The experimental results show that under a survey of 219 lung cancer chemotherapy patients with negative emotions and QoL satisfaction after chemotherapy, at a significance level of =  0.05, there is a linear regression relationship between mental resilience and anxiety and depression.

## 1. Introduction

Quality of Life (QoL) is a key thing to human health. Compared with other cancers, lung cancer ranks first in the incidence and mortality rate. It may be closely related to the increasing environmental pollution. According to World Health Organization (WHO) report, more than 1.1 million people die from lung cancer each year. Research data have shown that in the next 20 years, China will become the largest country with lung cancer, and the number of cases will increase year by year. From the analysis of the pathological types of lung cancer, the most common clinical-pathological type of lung cancer is non small cell lung cancer (NSCLC), and more than 80% of diagnosed cases are NSCLC. This pathological type of lung cancer is characterized by the absence of obvious pathological symptoms and clinical manifestations in early patients, and it has developed into clinical practice when the diagnosis is found.

RETRACTED

Advances in lung cancer medicine and diagnosis and treatment have prolonged the survival period of lung cancer patients. The impact of lung cancer on patients not only occurs physically, but also affects patients, their families, and society. This impact includes many aspects of the patient's physical, psychological and social functions. During chemotherapy, the patient not only suffers from the pain caused by the disease itself, but also suffers from the side effects of chemotherapy, such as nausea, vomiting, fatigue, and hair loss. These reactions can stimulate the patient's bad mood and affect the patient's QoL. China's research on the QoL of patients with lung cancer chemotherapy mainly focuses on new drugs, new therapies, the medical integration of Chinese and western medicines on cancer patients, and the relationship between radiotherapy and chemotherapy and the 5-year survival rate. However, there are few studies on the emotional and social support of lung cancer patients undergoing chemotherapy. A survey of patients' satisfaction with negative emotions and QoL after lung cancer chemotherapy shows that the cognitive behavioral therapy in this group can promote trauma, promote post-traumatic stress disorder and develop into injury, and help determine which factors can cause accidental trauma. The active psychological coordination for clinical nurses can provide a more reliable basis.

The rest of this paper is organized as follows: Section 2 discusses related work. A multi-modal behavior feature fusion model is constructed based on Coupled Hidden Markov Model (CHMM) in Section 3. The results are shown and discussed in Section 4.  Section 5 concludes this work.

## 2. Related Work

In the European Union, AI software that is correctly classified as a medical device must comply with rules that seek to establish its safety and performance [1]. Despite three rounds of multi-drug chemotherapy, the cancer is still developing despite the use of checkpoint inhibitors for treatment. When checkpoint inhibitors are no longer effective, mifepristone therapy can provide a way to stop metastatic lung cancer that is positive for PD-L1 markers [2]. The study found that distress thermometers can measure emotional problems and may have similarities in health-related QoL. Therefore, the study aimed to retrospectively evaluate the prognostic value of distress thermometers in lung cancer patients undergoing chemotherapy. This study included patients with stage III lung cancer who received carboplatin-containing chemotherapy in the Day Oncology Department from 2009 to 2014 and performed a distress thermometer in the first chemotherapy cycle [3]. Although the research perspective is forward-looking, there are still many unachievable parts of the technology.

RETRACTED

Based on coupled hidden markov model (CHMM), a multi-modal behavior feature fusion model was constructed to realize the understanding of human emotional intention in interactive activities [4, 5]. It had the following two main features.

1. First of all, there is a correlation between the changes in the expressions and physical behaviors of the interactors in the interactive behavior. Therefore, based on the modeling of the sequence in time, the correlation is also divided in space to extract differences. And the sequence of behaviors is handled separately [6].
2. Based on CHMM to model the problem, in the model, not only the different parts of the interaction behavior are modeled through each hidden Markov model (HMM) model, but also the relationship between multiple HMM models are modeled, thus fully showing the characteristics of the interaction behavior [7, 8].

The constructed a fusion model that mainly regards the facial expressions and body behaviors of the participants in the interaction as interrelated sequences and fusions them. In fusion, the model must not only fully express the characteristics of each sequence, but also must enable the relationship between the sequences to be expressed as in [9, 10, 11].

In maximum likelihood estimation, the difference from the HMM model is the belief propagation in the hidden state probability; and the maximization equation of the observation model is exactly the same as HMM model [12, 13]. In the fusion model based on the CHMM structure, there are mainly three hidden Markov chains. That is the facial expression sequence of the two interactors and the body action sequence in the interaction. Between these three sets of sequences, there is a mutual influence [14]. These three image sequences will be respectively used as the input observation sequence of the three hidden Markov chains in the constructed CHMM model to train the model [15].

## 3. Feature Fusion Based on CHMM

CHMM is a multi-dimensional extension of the hidden Markov model, which is shown in Figure 1.

In Figure 1, the current state not only depends on the previous state in the sequence M where it is located but also depends on the previous state in the other sequence N. This model has been widely used in computer vision and digital communications.

### 3.1. Parameter Estimation

In a CHMM containing two state sequences, *O*={*A*_1_^*T*^, *B*_1_^*T*^} represents an observation sequence, where *A*_1_^*T*^={*a*_1_,…, *a*_*T*_} represents the first observation sequence; similarly, *B*_1_^*T*^={*b*_1_,…, *b*_*T*_} represents the second observation sequence. *S*={*X*_1_^*T*^, *Y*_1_^*T*^} is a sequence of states, where *X*_1_^*T*^={*x*_1_,…, *x*_*T*_} represents the state of the first sequence; similarly, *Y*_1_^*T*^={*y*_1_,…, *y*_*T*_} represents the second sequence [16]. In addition, *P*(*M*_*t*+1_|*M*_*t*_,*N*_*t*_) is the state transition probability of the first sequence, and *P*(*N*_*t*+1_|*M*_*t*_,*N*_*t*_) is the state transition probability of the second sequence. *P*(*M*_1_) and *P*(*N*_1_) represent the initial probabilities of the first and second sequences, respectively. *P*(*A*_*t*_|*M*_*t*_) and *P*(*B*_*t*_|*N*_*t*_) represent the observation density of the two sequences, respectively. Here, for continuous time series, it is defined as a mixture of Gaussians, and *μ*_*x*_ and *μ*_*y*_ are defined as the mean, and ∑*x* and ∑*y* are the oblique variance matrices. *K*_*x*_ and *K*_*y*_ are the dimensional state spaces [17, 18], respectively.

RETRACTED

Based on the above parameter definitions, the likelihood probability of CHMM is expressed as follows:

(1) $$\begin{array}{c} L\left(\theta \right)=P\left(M_{1}\right)P\left(N_{1}\right)\overset{T}{\underset{t=1}{\prod }}P\left(A_{t}|M_{t}\right)P\left(B_{t}|N_{t}\right)B_{t}\text{.} \end{array}$$

*P*(*M*_*t*+1_|*N*_*t*_, *N*_*t*_)*P*(*N*_*t*+1_|*M*_*t*_, *N*_*t*_)*B*_*t*_|*N*_*t*_ In which, the vector contains parameters such as transition probability, initial probability, and observation density [19].

### 3.2. Maximum Likelihood Parameter Estimation

In this section, only the forward and backward recursive derivation of CHMM is introduced.

For the standard HMM model, the previous recursive process is as follows:

(2) $$\begin{array}{c} \alpha_{t+1}={P\left(A\right.}_{1}^{t+1},B_{t+1}=P\left(A_{t+1}|,|B_{t+1}\right)=P\left(A_{t+1}|,|B_{t+1}\right)\int \left.{PA}_{1}^{t},B_{t}\right)P\left(B_{t+1}|||B_{t}\right)dB_{t},\\ =P\left(A_{t+1}|B_{t+1}\right)\int P\left(B_{t+1}|B_{t}\right)dB_{t},\\ =P\left(A_{t+1}|B_{t+1}\right)P\left(B_{t+1}|A_{1}^{t+1}\right). \end{array}$$

In which, the corresponding variables A and B are defined for each sequence.

When *t* is equal to one, then we can get two equations as follows:

(3) $$\begin{array}{c} \begin{array}{c} \alpha_{t}^{A}=P\left(A_{1}|M_{1}\right)P\left(M_{1}\right),\\ \alpha_{t}^{B}=P\left(B_{1}|N_{1}\right)P\left(N_{1}\right). \end{array} \end{array}$$

In order to construct the CHMM model to realize the intention analysis based on the expression and body behavior in the interaction process, the hidden Markov chain and the relationship between them are defined as follows.

RETRACTED

### 3.3. Parameter Estimation

In this model, three hidden Markov chains are constructed. HMM-F1 and HMM-F2 are the expression sequences *φ*_*F*1_ and *φ*_*F*2_ modeling of the two interactors respectively, and HMM-B is the interactive motion sequence *φ*_*B*_ of the limbs. Assuming that there are N hidden states in each HMM, the hidden states are represented as *S*={*M*^*T*^, *N*^*T*^, *Z*^*T*^}, where *M*^*T*^={*x*_1_,…, *x*_*T*_} represents the state of the first sequence; similarly, *N*_1_^*T*^={*y*_1_,…, *y*_*T*_} represents the second sequence, and *Z*_1_^*T*^={*Z*_1_,…, *Z*_*T*_} is the state of the third sequence. *O*={*A*^*T*^, *B*^*T*^, *C*^*T*^} represents the observation sequence, where *A*^*T*^={*a*_1_,…, *a*_*T*_} represents the first observation sequence. *B*^*T*^={*b*_1_,…, *b*_*T*_} represents the second observation sequence, and *C*^*T*^={*c*_1_,…, *c*_*T*_} represents the third observation sequence. In addition, it is defined that P(*M*_*t*+1_|*M*_*t*_,*N*_*t*_, *Z*_*t*_) represents the state transition probability of the first sequence, P(*N*_*t*+1_|*M*_*t*_,*N*_*t*_, *Z*_*t*_) represents the state transition probability of the second sequence, and P(*Z*_*t*+1_|*M*_*t*_) represents the state transition probability of the third sequence. P(*M*_1_), P(*N*_1_), and P(*Z*_1_) represent the initial probabilities of the three sequences, respectively. P(*A*_1_|*M*_*t*_), P(*B*_1_|*N*_*t*_), and P(*C*_1_|*Z*_*t*_) represent the observation density of the three sequences, respectively. Based on the above parameter definitions, the model can be expressed as *γ*^*CHMM*^ = (M, N, Z, *π*), and the likelihood probability of CHMM is expressed as follows:

(4) $$\begin{array}{c} L\left(\theta \right)=P\left(M_{1}\right)P\left(N_{1}\right)P\left(Z_{1}\right)\prod_{t=1}^{T}P\left(A_{t}|M_{t}\right)P\left(B_{t}|N_{t}\right)P\left(C_{t}|Z_{t}\right),\\ \cdot P\left(M_{t+1}|M_{t},N_{t},Z_{t}\right)P\left(N_{t+1}|M_{t},N_{t},Z_{t}\right)P\left(Z_{t+1}|M_{t},N_{t},Z_{t}\right). \end{array}$$

### 3.4. Maximum Likelihood Parameter Estimation

The training of the model is realized by derivation based on the three HMM models. The derivation is based on the derivation of the preceding and following items proposed in the HMM model, and the specific process is as follows.

First, the training of each HMM model can be completed by the following formula, taking the first sequence as an example.

(5) $$\begin{array}{c} \begin{array}{c} \bar{P\left(X_{t+1}|X_{t},Y_{t},{\;Z}_{t}\right)}=\frac{\overset{T-1}{\underset{t=1}{\sum }}\left.\alpha_{t}\left(i\right)P\left(X_{t+1}\right)\left|X_{t},Y_{t},{\;Z}_{t}P\left(A_{t}\right)\right|Y_{t}\beta_{t+1}\left(j\right)\right)}{\overset{T-1}{\underset{t=1}{\sum }}\alpha_{t}\left(i\right)\beta_{t}\left(j\right)},\\ \bar{P\left(A_{t}|X_{t}\right)}=\frac{\overset{T}{\underset{t=1,o_{t}=O_{k}}{\sum }}\left.\alpha_{t}\left(i\right)\beta_{t}\left(j\right)\right)}{\overset{T}{\underset{t=1}{\sum }}\alpha_{t}\left(i\right)\beta_{t}\left(j\right)}. \end{array} \end{array}$$

In which, *α*_t_ and *β*_t_ are the antecedents and subsequent variables at time *t*, and their derivation is also extended based on the HMM model, as shown below.

RETRACTED

For the CHMM model, the corresponding variables *α*_*t*_^*A*^, *α*_*t*_^**B**^, and *α*_*t*_^*C*^ are defined for each sequence. When *t* is equal to one, *α*_*t*_^*A*^, *α*_*t*_^**B**^, and *α*_*t*_^*C*^ can be shown as follows:

(6) $$\begin{array}{c} \alpha_{1}^{A}=P\left(A_{1}|M_{1}\right)P\left(M_{1}\right),\\ \alpha_{1}^{B}=P\left(B_{1}|N_{1}\right)P\left(N_{1}\right),\\ \alpha_{1}^{C}=P\left(C_{1}|Z_{1}\right)P\left(Z_{1}\right). \end{array}$$

Other under the conditions of known *M*_2_, we can define *α*_2_^*A*^ as follows:

Since *A*_1_ and *A*_2_ are independent of each,

(7) $$\begin{array}{c} \alpha_{2}^{A}=P\left(A_{1}^{2}{,B}_{1}C_{1},M_{2}\right)\text{.} \end{array}$$

Thus, for any time *t*, repeat the above calculation, then we can get the following equations:

(8) $$\begin{array}{c} \begin{array}{c} \alpha_{t+1}^{A}=P\left(A_{t+1}|M_{t+1}\right)\iint \alpha_{t}^{A}\alpha_{t}^{B}\alpha_{t}^{C}P\left(M_{t+1}|M_{t},N_{t},Z_{t}\right)dM_{t}dN_{t}dZ_{t},\\ \alpha_{t+1}^{B}=P\left(B_{t+1}|N_{t+1}\right)\iint \alpha_{t}^{A}\alpha_{t}^{B}\alpha_{t}^{C}P\left(N_{t+1}|M_{t},N_{t},Z_{t}\right)dM_{t}dN_{t}dZ_{t},\\ \alpha_{t+1}^{C}=P\left(C_{t+1}|Z_{t+1}\right)\iint \alpha_{t}^{A}\alpha_{t}^{B}\alpha_{t}^{C}P\left(Z_{t+1}|M_{t},N_{t},Z_{t}\right)dM_{t}dN_{t}dZ_{t}. \end{array} \end{array}$$

Based on the derivation of the latter term in the HMM model, the derivation process of the latter term in the CHMM can be obtained as follows:

(9) $$\begin{array}{c} \begin{array}{c} \beta_{t+1}=P\left(O_{t+1}^{A}|S_{t}\right),\\ =\iint P\left(A_{t+1}|M_{t+1},N_{t+1},Z_{t+1}\right)P\left(B_{t+1}|M_{t+1},N_{t+1},Z_{t+1}\right)P\left(C_{t+1}|M_{t+1},N_{t+1},Z_{t+1}\right). \end{array} \end{array}$$

Based on the definition of the training derivation process of the above CHMM model, the specific algorithm is shown in (10) and (11).

(10) $$\begin{array}{c} \mu =\frac{\overset{K}{\underset{i=1}{\sum }}P\left({Seq}_{i}|CHMM\right)}{K}\text{,} \end{array}$$

(11) $$\begin{array}{c} \sigma =\sqrt{\frac{1}{K}\overset{K}{\underset{i=1}{\sum }}P\left({Seq}_{i}|CHMM\right)-\mu }\text{.} \end{array}$$

In which, *K* is the total number of training sequences, the average value represents the centroid of the CHMM model, and the standard deviation *σ* represents the radius of the CHMM model.

RETRACTED

## 4. Experiments of Negative Emotions and QoL Satisfaction Survey

### 4.1. General Information of Lung Cancer Patients Undergoing Chemotherapy

The age of the advanced patients in this group is 29–84 years old, with an average age of 55.65 ± 10.37 years old. Males account for the majority, and the male-female ratio is 2.17 : 1. All patients are advanced patients (II b: invasion of nearby important organs, IV: distant metastasis), and the pathological type is non-small cell lung cancer. Demographic data of lung cancer patients undergoing chemotherapy are shown in Table 1.

It can be seen from Table 1 that most patients (63.9%) have a lower-middle monthly family income (≤6000 yuan/month). Medical insurance patients account for 54.8%. Patients receive 2–6 courses of chemotherapy. The average number of chemotherapy courses is 3.34. After chemotherapy, the disease progresses 44 (20.1%), and the disease does not progress (including complete remission, partial remission, and stable disease) 175 (79.9%).

### 4.2. QoL of Lung Cancer Patients Undergoing Chemotherapy

Compared with the reference value (hereinafter referred to as the reference value) of the European Organization for Research and Treatment of Cancer (EORTC) survey of 1313 patients with stage II-IV lung cancer, the European Organization for Research and Treatment of Cancer-Quality of Life Questionnaire-Core-30 (EORTC-QLQ-C30) evaluates the overall QoL of this group of patients before chemotherapy. It can be seen from the score of the QoL: before chemotherapy, the patients in the group have the highest cognitive function scores and the lowest social function scores. The social function scores are lower Transthyretin value (TTRV) (*P* < 0.01), and the emotional (*P* < 0.05), physical, and role function scores are higher TTRV (*P* < 0.01). The results of analyzing the symptom dimensions show that the order of fatigue, pain, nausea, and vomiting before chemotherapy in this group is the same as the order of the reference value, but fatigue is lower TTRV (*P* < 0.01). The score order of the individual symptoms and the order of the reference value are similar, and the overall symptoms are milder TTRV. Among them, dyspnea and insomnia symptoms are significantly different from the reference value symptoms (*P* < 0.01). The financial difficulty score is higher TTRV (*P* < 0.01). EORTC-QLQ-C30 evaluation of the QoL of patients with lung cancer is shown in Table 2.

As shown in Table 2, the analysis of variance compares the QoL of lung cancer patients before and after chemotherapy. The results show that physical function, role function, cognitive function, and social function decline in the functional dimension (*P* < 0.01). The overall QoL decreases significantly (*P* < 0.01). However, it can be seen from the specific values that there is a big difference between before chemotherapy and during chemotherapy, before and after chemotherapy, and the difference between chemotherapy and after chemotherapy is small.

RETRACTED

Compared with the reference value (hereinafter referred to as the reference value) used to evaluate the QoL of 1313 patients with stage I to IV lung cancer with the special scale European Organization for Research and Treatment of Cancer-Quality of Life Questionnaire-Core-13 (EORTC-QLQ-L13) for lung cancer, this group of lung cancer patients has dyspnea, hair loss, arm, and shoulder pain before chemotherapy. The pain is milder (*P* < 0.01). EORTC-QLQ-LC13 evaluation of the QoL of patients with lung cancer is shown in Table 3.

As shown in Table 3, the analysis of variance compares the QoL of lung cancer patients before and after chemotherapy. The results show that treatment-related side effects, dysphagia, and degeneration are significantly increased (*P* < 0.01), and there is no significant difference in other symptoms (*P* > 0.05). The specific values showed cough symptom is alleviated.

### 4.3. Classification and Evaluation of the QoL of Patients with Lung Cancer Chemotherapy

EORTC-QLQ-C30 items are classified into three categories: functional dimension, overall QoL, and symptom dimension. EORTC-QLQ-LC13 is classified into two categories of lung cancer symptoms and lung cancer treatment-related side effects. The classification and comparison of the QoL before, during, and after chemotherapy measured by EORTC-QLQ-C30 and EORTC-QLQ-LC13 are shown in Table 4.

The classification and comparison of the QoL before, during, and after chemotherapy are shown in Figure 2.

It is clearly evident from Figure 2 that the scores of functional dimensions decrease significantly. That is, the patients' sensory function decreases. The scores of symptom dimensions increase significantly which means the clinical symptoms become more obvious, and the scores of side effects related to lung cancer treatment significantly. The side effects of chemotherapy increase significantly, and the overall QoL score decreases significantly (*P* < 0.01). The specific symptoms of lung cancer are relieved after chemotherapy.

Longitudinal studies on the correlation between coping style and QoL of patients with lung cancer chemotherapy divide the patients into the non-progressive group and the advanced group according to the efficacy of chemotherapy. The QoL of patients who does not progress after chemotherapy is compared with the overall QoL before chemotherapy. The comparison of the QoL between those who have not progressed and those who have progressed after chemotherapy is shown in Table 5.

RETRACTED

The classification and comparison of the QoL of patients with disease progression are shown in Figure 3.

Patients whose diseases do not progress after chemotherapy have poorer functional dimensions (*P* < 0.01), indicating that the patient's function has not returned to the level before chemotherapy. The scores of symptom dimensions and treatment-related side effects are significantly higher than those before chemotherapy (*P* < 0.01), indicating that the patients still have symptoms during and after chemotherapy, and treatment-related side effects are more obvious than those before chemotherapy. There is no statistically significant difference in overall QoL, lung cancer symptoms and before chemotherapy in patients who have not progressed after chemotherapy (*P* > 0.05). Comparing patients with non-progressed disease after chemotherapy and patients with the progressed disease, it is found that the QoL is significantly different in all dimensions, and the QoL of patients with the non-progressed disease is better than those with advanced disease (*P* < 0.01). Those who have not progressed after chemotherapy has milder symptoms and side effects.

### 4.4. QoL of Patients with Lung Cancer Chemotherapy

The differences in the QoL of patients with different curative effects by analysis of variance show that patients with different therapeutic effects after chemotherapy have significant differences in QoL (*P* < 0.01). Patients with good therapeutic effects have better functions and better overall QoL. The symptoms are mild, and the side effects related to treatment are also mild. The impact of chemotherapy on the QoL is shown in Table 6.

As shown in Table 6, the QoL decreases during chemotherapy. This study investigates the three-stage QoL of patients before chemotherapy (baseline), during chemotherapy (after the first intermittent period of chemotherapy), and after chemotherapy (after the last intermittent period of chemotherapy). The possible reasons for the decline in QoL are the patient's disease progression, the accumulation of toxicity of chemotherapy drugs, and so on. Chemotherapy for advanced lung cancer is only palliative treatment, and the possibility of a radical cure is extremely small. Some patients are ineffective in treatment. Disease progression or chemotherapy leads to toxicity. Longitudinal studies on the correlation between coping styles and QoL in patients with lung cancer should make it intolerable. As a result, the functional dimension of the patient's QoL decreases. Due to the lack of high specificity of current chemotherapy drugs, it kills tumor cells and at the same time damages, the body's normal cells, especially the fast-proliferating epithelial cells. Important organs will appear in patients receiving chemotherapy.

RETRACTED

The changing trends of various areas of the QoL of patients with lung cancer after chemotherapy with the course of treatment are shown in Figure 4.

It can be seen from Figure 4 that the QoL of lung cancer patients is worst before and after chemotherapy, best after the second chemotherapy, and reaches a downturn after the fourth and fifth chemotherapy, and then gradually improves. The normal situation is the worst after the surgery before chemotherapy, the best after the second chemotherapy, the lowest after the fourth chemotherapy, and then it improves. Social/family status usually declines gradually until the sixth chemotherapy improves. The emotional state is the worst after the surgery before chemotherapy, the best after the second chemotherapy, and the trend of improvement thereafter: the functional status is the worst after the surgery before chemotherapy and improves afterward.

### 4.5. Correlation Analysis of Coping Style and QoL after Chemotherapy

Pearson correlation is used to analyze the correlation between coping style and QoL after chemotherapy. The results of the correlation analysis of patients' coping style and QoL after chemotherapy are shown in Table 7.

As shown in Table 7, the positive coping style dependence on self is positively correlated with overall QoL (*P* < 0.01). Seeking support, facing positively, and covering up coping styles are positively correlated with the side effects of lung cancer treatment. Negative coping styles, venting emotions, escape, and fate (reverse scoring) are positively correlated with symptom dimensions and lung cancer treatment-related side effects (*P* < 0.01), and negatively correlated with functional dimensions and overall QoL (*P* < 0.01). That is patients who use less negative coping styles after chemotherapy have good QoL functions, good overall QoL, mild symptoms, and small side effects of treatment.

## 5. Conclusions

According to this study, it is necessary to improve the QoL of patients and the satisfaction of medical staff, and clinical staff should take some intervention measures for lung cancer patients undergoing chemotherapy. First of all, a comprehensive nursing evaluation is required to fully understand the physical, psychological, and social, common symptoms, side effects, and specific symptoms of lung cancer patients undergoing chemotherapy. It is recommended to use QoL as an indicator, and it will significantly affect the lives of lung cancer patients undergoing chemotherapy. The demographic and disease-related factors in quality provide a more detailed and targeted basis for formulating nursing measures. In addition, during the treatment of patients with lung cancer chemotherapy, it is recommended to evaluate the QoL of the patients as a comprehensive index for evaluating the impact of nursing interventions. The introduction of QoL into the medical world begins with tumor chemotherapy. Studies have shown that the use of different treatment options will not change the survival time of patients. Therefore, how to improve treatment during the survival period becomes the main topic of clinical research. In practice, the scale can not only assess the efficacy and risk of lung cancer treatment but also can conduct detailed and systematic studies throughout the life of the patient, providing a scientific basis for treatment and health care.

RETRACTED

## Figures and Tables

**Figure 1:** CHMM.

**Figure 2:** Classification and comparison of the QoL before, during and after chemotherapy measured by EORTC-QLQ-C30 and EORTC-QLQ-LC13 (mean).

**Figure 3:** Classification and comparison of the QoL of patients with disease progression after chemotherapy and those without disease progression after chemotherapy.

**Figure 4:** Trends in various areas of the QoL of patients with lung cancer after chemotherapy with the course of treatment.

**Table 1:** Demographic data of lung cancer patients undergoing chemotherapy (*n* = 219).

Category	Grouping	Number of cases	Composition ratio (%)
Sex	Male	139	63.5
	Female	80	36.5

Family income (month)	Below 3000 yuan	55	25. l
	3000–6000 yuan	85	38.8
	6000 yuan or more	79	36.1

Medical expenses	Own expense	75	34.2
	Medical insurance	120	54.8
	Other	24	4.0

Disease stage	III b	70	11.0
	IV	147	67.1

Chemotherapy effect	Totally relaxed	3	1.3
	Partial relief	66	30.1
	Stable disease	104	47.5
	Disease progression	44	20.1

**Table 2:** EORTC-QLQ-C30 evaluation of the QoL of patients with lung cancer ($\bar{X}\pm s$).

QLQ-C30	EORTC phase III-IV reference value (*n* = 1313)	Pre-chemotherapy score (*n* = 219)	*T* value	Post-chemotherapy score (*n* = 212)	*F* value
Cognitive function	85.3 ± 2.01	78.73 ± 19.74	−1.23	72.35 ± 22.09	4.89^*∗∗*^
Social function	68.8 ± 29.3	58.78 ± 26.31	−5.65^*∗∗*^	49.33 ± 31.83	5.76^*∗∗*^
Emotional function	67.3 ± 24.1	70.77 ± 21.66	2.28^*∗*^	67.75 ± 25.79	0.87
Physical function	64.9 ± 25.6	70.28 ± 23.86	2.60^*∗∗*^	56.63 ± 27.29	8.75^*∗∗*^
Role function	53.5 ± 31.3	63.52 ± 28.70	4.03^*∗∗*^	52.45 ± 32.74	8.20^*∗∗*^
Tired	43.2 ± 25.5	36.78 ± 19.96	−4.93^*∗∗*^	45.72 ± 25.69	10.23^*∗∗*^
Pain	34.5 ± 31.7	29.31 ± 21.85	−3.24^*∗∗*^	35.17 ± 28.56	3.00^*∗*^
Feel sick and vomit	10.8 ± 19.1	15.11 ± 22.35	2.74^*∗∗*^	24.00 ± 24.93	10.64^*∗∗*^
Insomnia	34.7 ± 33.4	27.42 ± 24.33	−4.26^*∗∗*^	46.67 ± 31.53	28.12^*∗∗*^
Difficulty breathing	40.7 ± 32.2	31.86 ± 25.97	−4.85^*∗∗*^	30.00 ± 30.08	0.67
Loss of appetite	31.1 ± 24.6	27.75 ± 27.38	−1.74	41.17 ± 23.26	12.51^*∗∗*^
Constipation	22.2 ± 21.7	19.38 ± 16.05	−1.54	31.17 ± 33.26	7.84^*∗∗*^
Financial difficulties	14.0 ± 24.3	48.75 ± 35.61	14.08^*∗∗*^	60.50 ± 35.38	4.81^*∗∗*^
Diarrhea	7.1 ± 8.3	7.88 ± 6.36	0.51	10.33 ± 9.88	0.92

RETRACTED

**Table 3:** EORTC-QLQ-LC13 evaluation of the QoL of patients with lung cancer ($\bar{X}\pm s$).

QLQ-LC13	EORTC phase III-IV reference value (*n* = 1313)	Pre-chemotherapy score (*n* = 219)	*T* value	Post-chemotherapy score (*n* = 212)	*F* value
Cough	38.4 ± 22.3	35.47 ± 23.14	−1.78	32.76 ± 23.54	0.92
Hemoptysis	7.7 ± 17	12.64 ± 13.54	3.70^*∗∗*^	14.33 ± 21.27	0.39
Difficulty breathing	21.5 ± 24.6	25.34 ± 21.37	−4.14^*∗∗*^	28.06 ± 25.08	1.26
Mouth pain	5.1 ± 14.9	11.00 ± 18.24	4.45^*∗∗*^	13.24 ± 22.39	1.69
Hard to swallow	6.8 ± 17.8	10.02 ± 20.35	2.20^*∗*^	15.33 ± 26.09	4.89^*∗∗*^
Peripheral neuralgia	8.9 ± 19.36	15.60 ± 23.11	4.10^*∗∗*^	21.00 ± 28.17	2.47
Hair loss	5.2 ± 19.17	1.15 ± 8.38	−6.89^*∗∗*^	37.50 ± 32.90	115.74^*∗∗*^
Chest pain	20.8 ± 26.6	25.94 ± 27.35	2.69^*∗∗*^	29.00 ± 30.50	0.72
Arm shoulder pain	22.4 ± 27.52	16.42 ± 24.42	−3.51^*∗∗*^	18.83 ± 27.27	1.76
Other pain	23.8 ± 13.4	18.06 ± 15.19	−3.45^*∗∗*^	20.67 ± 17.81	1.66

**Table 4:** Classification and comparison of the QoL before, during and after chemotherapy measured by EORTC-QLQ-C30 and EORTC-QLQ-LC13 ($\bar{X}\pm s$).

QoL dimension	Pre-chemotherapy score (*n* = 219)	During chemotherapy (*n* = 212)	Post-chemotherapy score (*n* = 212)	*F* value
Functional dimension	65.70 ± 12.28	59.74 ± 11.14	59.57 ± 17.38	42.56^*∗∗*^
Overall QoL	56.28 ± 17.32	55.09 ± 19.82	51.50 ± 20.18	12.13^*∗∗*^
Symptom dimension	27.26 ± 13.26	34.75 ± 12.04	36.19 ± 14.73	71 67^*∗∗*^
Lung cancer symptoms	22.31 ± 17.37	24.80 ± 15.76	23.16 ± 12.57	5.31^*∗∗*^
Related side effects	9.44 ± 7.23	20.77 ± 18.01	21.31 ± 13.34	34.32^*∗∗*^

**Table 5:** Comparison of the QoL between those who have not progressed and those who have progressed after chemotherapy.

QoL dimension	Pre-chemotherapy score (*n* = 219)	Post-chemotherapy (disease has not progressed) (*n* = 175)	*T*1 value	Post-chemotherapy (disease progression) (*n* = 44)	*T*2 value
Functional dimension	68.44 ± 16.28	63.52 ± 19.43	2.61	47.36 ± 23.09	4.52^*∗∗*^
Overall QoL	56.28 ± 21.32	54.49 ± 19.06	0.827	40.06 ± 20.66	4.30^*∗∗*^
Symptom dimension	27.73 ± 15.26	33.72 ± 17.94	−3.83^*∗∗*^	44.34 ± 18.28	−3.50^*∗∗*^
Lung cancer symptoms	22.31 ± 13.86	22.23 ± 9.37	0.05	30.95 ± 18.47	−2.83^*∗∗*^
Related side effects	9.44 ± 8.05	19.52 ± 13.15	−6.69^*∗∗*^	31.18 ± 22.43	−3.46^*∗∗*^

RETRACTED

**Table 6:** The effect of the efficacy of chemotherapy on the QoL (*n* = 212).

Influencing factors	Functional dimension	Symptom dimension	Overall QoL	Related side effects	Lung cancer symptoms
Treatment effect	10.73^*∗∗*^	11.90^*∗∗*^	10.73^*∗∗*^	6.39^*∗∗*^	5.47^*∗∗*^

**Table 7:** Correlation analysis of patients' coping style and QoL after chemotherapy (*r*) (*n* = 212).

Solution	Functional dimension	Symptom dimension	Overall QoL	Related side effects	Lung cancer symptoms
Optimism	0.06	−0.06	0.14	0.13	0.01
Self-reliance	0.04	−0.07	0.17^*∗∗*^	0.12	0.04
Seek support	−0.06	0.01	0.05	0.20^*∗∗*^	0.08
Face positively	−0.02	−0.01	0.06	0.17^*∗∗*^	0.12
Cover up	0.05	−0.01	0.11	0.16^*∗∗*^	0.13
Vent emotions	0.19^*∗∗*^	−0.21^*∗∗*^	0.22^*∗∗*^	−0.26^*∗∗*^	−0.19^*∗∗*^
Escape	0.14	−0.17^*∗∗*^	0.11	−0.28^*∗*^	−0.23^*∗∗*^
Fate	0.19^*∗∗*^	−0.23^*∗*^	0.15^*∗*^	−0.29^*∗∗*^	−0.17^*∗∗*^

## Data Availability

The simulation experiment data used to support the findings of this study are available from the corresponding author upon request.
